The article "Novel Role of Phosphorylation-Dependent Interaction between FtsZ and FipA in Mycobacterial Cell Division" was retracted in 2022. Reasons: manipulated images; duplicated images; original data or images not available; unreliable results or conclusions.

# Novel Role of Phosphorylation-Dependent Interaction between FtsZ and FipA in Mycobacterial Cell Division

**DOI:** 10.1371/journal.pone.0008590

**Published:** 2010-01-06

**Authors:** Kamakshi Sureka, Tofajjen Hossain, Partha Mukherjee, Paramita Chatterjee, Pratik Datta, Manikuntala Kundu, Joyoti Basu

**Affiliations:** Department of Chemistry, Bose Institute, Kolkata, India; University of Hyderabad, India

## Abstract

The bacterial divisome is a multiprotein complex. Specific protein-protein interactions specify whether cell division occurs optimally, or whether division is arrested. Little is known about these protein-protein interactions and their regulation in mycobacteria. We have investigated the interrelationship between the products of the *Mycobacterium tuberculosis* gene cluster *Rv0014c-Rv0019c*, namely PknA (encoded by *Rv0014c*) and FtsZ-interacting protein A, FipA (encoded by *Rv0019c*) and the products of the division cell wall (*dcw*) cluster, namely FtsZ and FtsQ. *M. smegmatis* strains depleted in components of the two gene clusters have been complemented with orthologs of the respective genes of *M. tuberculosis*. Here we identify FipA as an interacting partner of FtsZ and FtsQ and establish that PknA-dependent phosphorylation of FipA on T77 and FtsZ on T343 is required for cell division under oxidative stress. A *fipA* knockout strain of *M. smegmatis* is less capable of withstanding oxidative stress than the wild type and showed elongation of cells due to a defect in septum formation. Localization of FtsQ, FtsZ and FipA at mid-cell was also compromised. Growth and survival defects under oxidative stress could be functionally complemented by *fipA* of *M. tuberculosis* but not its T77A mutant. Merodiploid strains of *M. smegmatis* expressing the FtsZ(T343A) showed inhibition of FtsZ-FipA interaction and Z ring formation under oxidative stress. Knockdown of FipA led to elongation of *M. tuberculosis* cells grown in macrophages and reduced intramacrophage growth. These data reveal a novel role of phosphorylation-dependent protein-protein interactions involving FipA, in the sustenance of mycobacterial cell division under oxidative stress.

## Introduction

Cell growth and division involves exquisite temporal and spatial regulation of a succession of events which include choice of the site of division, positioning of the Z-ring at mid-cell, and formation of the septum [1]–[3]. The fidelity of cell division occurring at mid-cell depends on the assembly of a macromolecular complex at the site of division involving recruitment of proteins in a hierarchial manner [4]–[6]. In most Gram-negative and Gram-positive bacteria, genes whose products are involved in cell division, cluster in a chromosomal region termed the *dcw* (division and cell wall) cluster [7]. The principal player in driving cytokinesis is FtsZ, a GTP-binding protein considered to be the bacterial counterpart of eukaryotic tubulin [8], [9]. It is encoded by a gene within the *dcw* cluster. It forms the Z-ring [10] which serves as a cytoskeletal scaffold for the sequential recruitment and assembly of the multiprotein complex that comprises the divisome [11], [12]. Mycobacteria share many components of the cell division machinery identified in other bacteria. However, it is likely that there are several unique features in the mechanism of cell division in mycobacteria, considering that assisters of Z ring formation such as FtsA and ZipA have not been identified, nor have counterparts of the MinCD system which ensures that division occurs at midcell. For example, it is possible that direct interaction between FtsZ and FtsW stabilizes FtsZ at the membrane and links cell division to septal peptidoglycan biosynthesis [13], [14].

A family of 11 serine/threonine protein kinases (STPKs) are likely sensors of environmental signals in mycobacteria [15], [16]. In spite of an interest in this family of kinases in recent years, there is limited understanding of the signals that they sense and the consequences of such sensing. The STPKs of mycobacteria with the exception of PknG and PknK, have extracellular C-terminal sensory domains and intracellular N-terminal kinase domains. Cell wall biogenesis, cell division, central metabolic processes such as the TCA cycle and gene expression, are among the growing body of processes that are regulated by STPK-mediated phosphorylation in mycobacteria [16]–[18].

Both PknA and PknB are involved in regulation of cell shape [19], [20]. These two kinases reside in a genomic region (encompassing the ORFs Rv0014c-Rv0019c in *Mycobacterium tuberculosis* H37Rv) that is conserved across all species of mycobacteria for which genome sequences are available. This region also encodes PstP, the cognate phosphatase of PknA and PknB; PBPA, a penicillin-binding transpeptidase [19], and RodA, a putative player in cell shape maintenance. PknA and PknB phosphorylate Wag31[20], and PknB phosphorylates PBPA (Dasgupta *et al*., 2006). A phosphorylation-defective mutant of PBPA fails to localize to the site of division. In *M. tuberculosis*, this conserved gene cluster containing morphogenetic genes, also harbours the genes *Rv0019c* and *Rv0020c*, encoding two forkhead-associated domain (FHA) proteins. The FHA domain is a phosphopeptide recognition motif spanning 80 to 100 amino acid residues folded in an 11-stranded beta sandwich which recognizes phosphopeptide [21], [22]. PknB phosphorylates Rv0020c *in vitro* [23]. As of now, the functional role of Rv0020c remains unclear.

Key to regulated cell division are proteins which inhibit or stabilize assembly of the divisome at mid-cell. In mycobacteria, some of the above findings have suggested that serine/threonine kinases such as PknA and PknB fine tune the process of cell division, and it is tempting to speculate that accessory proteins unique to mycobacteria, as well as dynamic protein phosphorylation could play vital roles in controlling cell septation, particularly under conditions of stress. We have tested the possibility molecular interactions among proteins encoded by genes of the *dcw* cluster and those encoded by the cluster *Rv0014c-Rv0019c* regulate cell division in mycobcteria. This report focuses on the forkhead-associated domain (FHA)-containing protein encoded by *Rv0019c*. A role for this gene product in cell division was tested by knocking out its counterpart in *Mycobacterium smegmatis*. The increased susceptibility of the mutant to oxidative stress and the altered cell morphology, further supported our contention that this particular FHA-domain-containing protein could regulate cell division. Using a variety of biochemical and genetic approaches, we demonstrate that in mycobacteria, FtsZ, FtsQ and the product of the ORF *Rv0019c*, form a ternary complex. In view of its ability to interact with FtsZ, we name this gene product, FtsZ-interacting protein A (FipA). The FipA-FtsZ interaction is dependent on PknA which phosphorylates FipA on amino acid residue T77 and FtsZ on T343. We demonstrate that knock down of *pknA* impairs the formation of the FtsZ-FtsQ-FipA complex. FtsZ fails to localize at mid-cell in *fipA* knock out *M. smegmatis* cells under oxidative stress and localization is rescued by complementation with FipA_MTB_. An important role of FipA is further suggested by the fact that depletion of FipA leads to reduced growth of *M. tuberculosis* in macrophages.

## Results

### Effect of Inactivation of FipA_MSMEG_ and Knock Down of FipA in *M. tuberculosis*

The genomic region encompassing the ORFs *Rv0014c* to *Rv0019c* (Figure S1A) of *M. tuberculosis*, is conserved across mycobacterial species. Its role in cell division and the function of some of the genes encoded by this region has been conjectured over the years. The genes *Rv0014c-Rv0018c* are organized in an operon. The ORF *Rv0016c* encodes PBPA, a transpeptidase that regulates cell morphology in a manner dependent on phosphorylation by the product of the ORF *Rv0014c*, PknB [19]. The product of the ORF *Rv0015c*, PknA phosphorylates Wag31 thereby regulating cell morphology [20]. *Rv0018c* encodes PstP, a phosphatase which dephosphorylates substrates such as phospho-PBPA. The function of FipA (the product of the adjacent transcriptional unit *Rv0019c*), a putative FHA protein, remains obscure. Computational analysis of genome-wide functional linkages, suggests that FipA has a role in cell envelope biosynthesis in *M. tuberculosis* [24]. Considering that FipA is conserved across pathogenic and non-pathogenic mycobacterial species, we chose *M. smegmatis*, the fast-growing non-pathogenic strain in order to understand the role of FipA in mycobacterial physiology. The deduced amino acid sequences of FipA_MSMEG_ and FipA_MTB_ (Figure S1B) show that the proteins are 88% identical in amino acid sequence. To test the role of FipA in cell growth and division, *fipA* was inactivated at its native locus in *M. smegmatis*. The absence of FipA was confirmed by Western blotting (Figure S2A). We also confirmed by Western blotting that the expression of PknB, PknA, PBPA and PstP encoded by neighboring genes, was not affected (Fig. S2A). The mutated strain will be referred to as FipA-KO. The morphology and the growth rates of wild type *M. smegmatis* mc^2^155 and FipA-KO were compared. FipA-KO exhibited reduced growth compared to the wild type in Middle Brook 7H9 broth supplemented with Tween 80. The wild type reached mid-log phase at 20 h, whereas the mutant reached mid-log phase at 24 h (Fig. 1A). At stationary phase, the growth of the mutant was lower than that of the wild type. Considering the lowered growth of the mutant particularly at stationary phase, we speculated that it was possibly less capable of handling stressful conditions than the wild type. We tested its susceptibility to conditions of stress. FipA-KO was more susceptible to H_2_O_2_ stress than the wild type (Fig. 1B). In order to test whether FipA is required for cell division under H_2_O_2_-induced oxidative stress, we determined cell lengths in the wild type and FipA-KO. In the absence of exogenous stress, cells of the wild type and FipA-KO were of similar length. However, approximately 40% of the cells were >6 µm in length in the knockout strain subjected to oxidative stress (Fig. 1C). In comparison, <5% of the wild type cells were >6 µm in length under similar oxidative stress. These results suggest that FipA is required to sustain cell division in bacteria subjected to oxidative stress. In order to assess the ability of FipA of *M. tuberculosis* to complement FipA-KO, a single copy of *fipA* of *M. tuberculosis* was integrated into the chromosome of FipA-KO. Complementation of FipA was confirmed by Western blotting (Fig. S2A). FipA-KO complemented with *fipA*_MTB_, was visualized by microscopy before and after subjecting to oxidative stress. Complementation with *fipA_MTB_* restored the cell length of FipA-KO to resemble that of the wild type (Fig. 1C). In addition, growth defect was rescued (Fig. 1A), and the complemented strain could withstand oxidative stress (Fig. 1B) to an extent similar to the wild type. This also confirmed that the difference in phenotypic behavior between the wild type and FipA-KO was attributable specifically to the absence of FipA.

**Figure 1:** FipA regulates growth and cell division. A. Growth of *M. smegmatis* mc^2^ 155 (WT), FipA-KO (KO) or FipA-KO complemented with *fipA*_MTB_ (WT) or its *fipA*_MTB(T77A)_ [complemented (T77A)], was followed by monitoring cfu at different periods of time. B. Cultures were treated with H_2_O_2_ as described under “Materials and Methods.” Growth was monitored by determining cfu. Percent survival was determined with respect to the cfu of untreated cells (100%). C. Cell length measurements of wild type *M. smegmatis* (WT), or FipA-KO (KO), or FipA-KO complemented with *fipA_MTB_* (complemented) after treatment with H_2_O_2_ as described under “Materials and Methods.” At least 100 cells from each set were measured. D. Western blotting of lysates of *M. tuberculosis* expressing an antisense construct of *fipA* under the control of the *hsp60* promoter, with anti-FipA antibody. The blot was reprobed with anti-FtsW as loading control. E. THP1 cells were infected with *M. tuberculosis* harbouring vector alone or an antisense construct of *fipA* at an MOI of 2 for 90 min; washed with fresh medium and grown for different periods of time. Internalized bacteria were released by lysing the macrophages followed by determination of cfu. *M. tuberculosis* harbouring vector alone, -▵-; or antisense construct of *fipA*, -•-. F, G. THP-1 cells were infected and intracellular bacteria were obtained by lysing the macrophages, as in (E). Cell length measurements were done for intracellular *M. tuberculosis* harbouring vector alone (F) or expressing an antisense construct of *fipA* under the control of the *hsp60* promoter (G) after 1, 3, 5, or 6 days of growth in THP1 cells. At least 100 cells from each set were measured.

The division defect occurring after H_2_O_2_ treatment in FipA-KO could possibly be due to induction of the SOS response. RecA and LexA are two principal proteins involved in the SOS response [25], [26]. We checked the transcription levels of *recA* and *lexA* after treatment with H_2_O_2_. No increase in *lexA* or *recA* was observed in either the wild type or FipA-KO or FipA-KO complemented with *fipA*_MTB_ (Figure S2B, C). O' Sullivan *et al.* [27] have reported that *recA* and *lexA* transcription increases after exposure of *M. tuberculosis* to mitomycin C, a compound that alkylates and crosslinks DNA and induces the SOS response. Mitomycin C exposure was therefore used as a positive control for induction of the SOS response. In this case, *recA* and *lexA* transcription increased in the wild type, FipA-KO and FipA-KO complemented with *fipA*_MTB_ (Figure S2B, C). Taken together, this suggests that the division defect in FipA-KO cells after H_2_O_2_ treatment is not due to induction of the SOS response.

In order to assess the role of FipA in *M. tuberculosis* growing in macrophages, we knocked down *fipA* of *M. tuberculosis* (Fig. 1D). This knock down compromised the ability of *M. tuberculosis* to multiply within macrophages after two days (Fig. 1E). This argued in favor of a role of FipA in mycobacterial multiplication in macrophages. A defect in cell division in the *fipA*-knocked down cells in macrophages was confirmed by the observation that the percentage of macrophage-grown cells over 6 µm in size was consistently higher in *fipA-* knocked down cells compared to the wild type over a period of 6 days (Fig. 1F, G). This suggests that FipA is required to sustain mycobacterial cell division in macrophages.

### FipA Interacts with FtsZ *In Vivo*

In view of the fact that FtsZ provides the driving force of cytokinesis by forming the Z-ring at the septum [1], and that knock out of *fipA* is associated with a septation defect, we tested the possibility that FtsZ and FipA are interacting partners *in vivo*. In order to analyze the interaction of FipA with FtsZ, FtsZ was immunoprecipitated from cell lysates of *M. tuberculosis* or *M. smegmatis*, and the presence of FipA in the immunoprecipitates was tested using anti-FipA antibody. FtsZ immunoprecipitates pulled down endogenous FipA (Fig. 2A). In order to understand the role of FHA domain in the interaction of FipA with FtsZ, FipA-KO was complemented with wild type *fipA_MTB_* or *fipA_MTB_* harboring mutations in conserved amino acid residues of the FHA domain encompassing amino acid residues P82 to V132. FHA domain mutants S101A, H104A and N123A of FipA were impaired in their ability to interact with FtsZ *in vivo* (Fig. 2B). On the other hand, the FipA (D118A) mutant retained the ability to interact with FtsZ. These results suggest that the FHA domain of FipA plays a role in its interaction with FtsZ *in vivo*.

**Figure 2:** The FHA domain of FipA is required for its interaction with FtsZ. A. Cell lysates of *M. tuberculosis* or *M. smegmatis* were immunoprecipitated (IP) with anti-FtsZ antibody and immunoblotted (IB) with anti-FipA antibody or antibody against an irrelevant protein (PPK1) [as a negative control]. The blot was reprobed with anti-FtsZ antibody to show equal loading. B. Lysates of *M. smegmatis* mc^2^155 or FipA-KO complemented with the wild type (WT) or different mutants of FipA_MTB_, were immunoprecipitated with anti-FipA antibody followed by immunoblotting with anti-FtsZ antibody and reprobing with anti-FipA antibody. Blots shown are representative of three separate experiments.

FHA domains are known to interact with ser/thr kinases [21]. Therefore, we tested whether FipA of *M. smegmatis* (FipA_MSMEG_, encoded by MSMEG_0034), is phosphorylated *in vivo*. FipA was immunoprecipitated from cell lysates of *M. tuberculosis* or *M. smegmatis* followed by Western analysis using anti-phosphothreonine antibody. The results affirmed that FipA_MTB_ and FipA_MSMEG_ are phosphorylated *in vivo* on threonine (Fig. 3A). Incubation of immunoprecipitates with purified PstP resulted in dephosphorylation of agarose-bound FipA_MTB_ and FipA_MSMEG_ (Fig. 3A). In a reverse experiment, capture of proteins from lysates of *M. smegmatis* on phosphothreonine agarose, followed by Western analysis of the bound proteins with anti-FipA antibody, also confirmed that FipA is phosphorylated within cells (Fig. 3B).

**Figure 3:** FipA is phosphorylated *in vivo* and localizes to the membrane. A, B. Lysates of *M. tuberculosis*(A) or *M. smegmatis* (A, B) were immunoprecipitated either with anti-FipA antibody (A) or with phosphothreonine agarose (B), left untreated (−) or treated (+) with S-tagged PstP_MTB_ followed by immunoblotting with anti-phosphothreonine (A) or anti-FipA (B) antibody as indicated; and reprobing with anti-FipA antibody for panel A. C. Cell lysates were fractionated and membrane and cytosolic fractions were immunoblotted with anti-FipA antibody followed by reprobing with anti-FtsZ (marker for the cytosol) or with anti-FtsW (membrane marker). Blots shown are representative of three separate experiments.

### Subcellular Localization of FipA

In order to understand the function of FipA and in view of the fact that it interacts with FtsZ, we felt it imperative to localize FipA in cells. Its topology predicted using the program HMMTOP [28] suggest that it is a transmembrane protein. Fractionation of lysates into membranes and cytosolic components, followed by Western blotting confirmed that FipA localizes in mycobacterial membranes (Fig. 3C). Crosscontamination of membrane and cytosol fractions was ruled out by the fact that membranes were positive for the membrane protein FtsW but not for the cytosolic protein FtsZ, whereas the cytosol fraction was positive for FtsZ but not for FtsW.

### FipA Is Phosphorylated by PknA

In order to test whether FipA is phosphorylated by the neighbouring ser/thr kinase PknA, we expressed FipA in *E. coli* with an N-terminal hexahistidine or S-tag. Purified His-tagged FipA migrated as a protein of approximately 20 kDa (Fig. 4A). We expressed and purified the kinase domain of PknA encompassing Y13 to A273 (PknA_13–273_) as a GST-tagged protein (Fig. 4B). Recombinant FipA could be phosphorylated by PknA_13–273_ in the presence of Mg^2+^ and [γ-^32^P] ATP (Fig. 4C). The kinase-dead K42A mutant of PknA_13–273_ [20] was unable to phosphorylate FipA (Fig. 4C). In order to evaluate the role of FHA domain amino acid residues S101, H104, D118 and N123 on interaction of FipA with PknA and its phosphorylaton, these residues were individuallly mutated to alanine. None of the mutants other than the D118A mutant, could interact with PknA_13–273_ (Fig. 4D), nor were these mutants (with the exception of D118A) phosphorylated by PknA (Fig. 4E). These results confirmed the importance of the FHA domain residues S101, H104, and N123 in interaction with PknA and in PknA-mediated phosphorylation of FipA.

**Figure 4:** FipA interacts with, and is phosphorylated by PknA *in vitro*. A, B. Coomassie blue-stained gels of uninduced (1), or induced (2) cells of *E. coli* expressing FipA (A), GST-PknA_13-273_ (B), purified FipA (A, lane 3) and GST-PknA_13–273_ (B, lane 3). C. Purified FipA was phosphorylated by GST-PknA_13–273_ or its K42A mutant *in vitro* in the presence of [γ-^32^P] ATP followed by autoradiography. D. Recombinant S-tagged FipA or its mutants were incubated with GST-PknA_13–273_ bound to glutathione-Sepharose beads. Proteins bound to the beads were detected by immunoblotting with anti-FipA antibody. The blot was reprobed with anti-GST antibody. E. Purified FipA or its mutants were phosphorylated by GST-PknA_13–273_ *in vitro* in the presence of [γ-^32^P] ATP followed by autoradiography. The first lane represents autophosphorylated GST-PknA_13–273_. Blots shown are representative of three separate experiments. Lower blots of panels C and E are Coomassie blue-stained gels showing the levels of FipA.

The NET Phos program [29] predicted threonine residues at positions 77 and 142 as putative phosphorylatable residues. Mutation of T77 abrogated PknA_13–273_-dependent phosphorylation of FipA, (Fig. 4E) but not its interaction with PknA (Fig. 4D). This identified T77 as a possible site of PknA-dependent phosphorylation. Mutation of T142 had no effect in PknA_13–273_-mediated phosphorylation (data not shown). In order to confirm that FipA is phosphorylated on a single threonine residue by PknA_13–273_, mass analysis of His-FipA and the protein phosphorylated by PknA_13-273_, was undertaken. The increase in the molecular mass of the intact protein (Figure S3), confirmed incorporation of a single phosphate residue by PknA_13–273_.

In order to investigate the role of phosphorylation of FipA on its interaction with FtsZ, FipA-KO was complemented with *fipA*_MTB_ or *fipA*_MTB(T77A)_. Wild type FipA_MTB_ could immunoprecipitate FtsZ (Fig. 2B) while the T77A mutant could not, suggesting the requirement of FipA phosphorylation for its interaction with FtsZ. In addition, phosphorylation-defective FipA(T77A) could not restore the growth defect of the FipA-KO (Fig. 1A) or its ability to withstand H_2_O_2_ stress (Fig. 1B). This suggests that phosphorylation of FipA on T77 is required to support survival under oxidative stress.

### FipA Is Phosphorylated *In Vivo* by PknA in Mycobacteria

In order to demonstrate PknA-dependent phosphorylation of FipA *in vivo,* we performed gradual depletion of the protein in *M. smegmatis* by acetamide-inducible expression of an antisense construct of *pknA*. Depletion of PknA was confirmed by immunoblotting of lysates with anti-PknA antibody (Fig. 5A). Gradual depletion of PknA was concomitant with gradual decrease in threonine phosphorylation of FipA (Fig. 5B), suggesting that PknA mediates phosphorylation of FipA *in vivo*.

**Figure 5:** A, B. FipA is phosphorylated *in vivo* in a PknA-dependent manner. A, B. *M. smegmatis* was transformed with a construct carrying *pknA* in antisense orientation under an acetamide-inducible promoter. Transformed cells were induced with 0.2% acetamide for the indicated periods of time in order to downregulate *pknA* expression. Antisensing was followed by immunoblotting of cell lysates with anti-PknA antibody, followed by reprobing with anti-FtsW antibody (A); or cell lysates at different periods of time were immunoprecipitated with anti-FipA antibody followed by immunoblotting with anti-phosphothreonine antibody and reprobing with anti-FipA antibody (B). Blots shown are representative of three separate experiments. IB: immunoblotting; IP: immunoprecipitation.

### Interaction of FtsZ with FipA Is Required for Septal Localization of FtsZ under Oxidative Stress

Considering that FipA interacts with FtsZ *in vivo* (Fig. 2), we attempted to understand whether this interaction is necessary for the localization of FtsZ at mid-cell in dividing cells. Immunolocalization of FtsZ in FipA-KO showed that FtsZ was compromised in its ability to localize at mid-cell in FipA-KO cells subjected to oxidative stress (Fig. 6A, B), but could localize to mid-cell in the absence of oxidative stress (data not shown). Complementation of FipA-KO with *fipA*_MTB_ restored the localization of FtsZ at mid-cell even under oxidative stress (Fig. 6C,D). The frequency of Z ring formation in the absence or presence of oxidative stress, was measured by microscopy. The data presented in Table 1 clearly indicate that Z ring formation under oxidative stress requires FipA. No Z ring formation could be observed in FipA-KO under oxidative stress. However, complementation with *fipA*_MTB_ restored Z ring formation in 63 out of 81 FtsZ-positive cells (Table 1). We hypothesize that FipA facilitates localization of FtsZ at mid-cell under H_2_O_2_ stress.

**Figure 6:** Localization of FtsZ to mid-cell in *M. smegmatis* under oxidative stress requires FipA. FipA-KO (A,B) or FipA-KO complemented with *fipA*_MTB_ (C, D) was subjected to stress by incubation in the presence of H_2_O_2_ as described under “Materials and Methods”. Immunolocalization of FtsZ was carried out by incubation with anti-FtsZ antibody followed by staining with Alexa 488-conjugated rabbit IgG (green). Images shown are fluorescence micrographs (A, C) and the merge of phase contrast and fluorescence micrographs (B,D). Bar, 2 µm.

**Table 1:** Presence of Z ring in cells.

	Total	septum	poles	others
WT without stress	122	102	18	2
WT after H_2_O_2_ stress	105	79	17	9
FipA-KO without stress	101	81	10	10
FipA-KO after H_2_O_2_ stress	-	-	-	-
FipA-KO complemented with *fipA*_MTB_ without stress	102	75	21	6
FipA-KO complemented with *fipA*_MTB_, after H_2_O_2_ stress	81	63	14	4

FtsZ positive cells were counted.

### PknA-Mediated Phosphorylation of FtsZ

The present study shows that FipA is phosphorylated by PknA on T77 (Fig. 4E) and phosphorylation is required for its interaction with FtsZ (Fig. 2B). Thakur and Chakraborti (2006) had earlier demonstrated that FtsZ is phosphorylated by PknA without identifying the site of PknA-dependent FtsZ phosphorylation. In order to further understand the role of PknA-dependent phosphorylations, we attempted to identify the site of phosphorylation of FtsZ. Computational analysis using the Net Phos program [29], suggested that T343 is a putative site of phosphorylation of FtsZ. Recombinant PknA_13–273_ could phosphorylate recombinant wild type His-FtsZ_MTB_ but not the T343A mutant *in vitro* (Fig. 7A). In addition, mass analysis of FtsZ_MTB_ after phosphorylation by PknA_13–273_ showed an increase in mass corresponding to phosphorylation on a single residue by (Figure S4). The T343A mutant, on the other hand, showed no increase in mass after treatment with PknA_13-273,_ supporting our contention that T343 represents the only site of PknA-mediated phosphorylation of FtsZ. In order to confirm PknA-mediated threonine phosphorylation of FtsZ *in vivo*, *pknA* was partially knocked down by inducing the expression of an antisense RNA to *pknA* driven by the acetamidase promoter. Knock down of *pknA* inhibited phosphorylation of FtsZ on threonine (Fig. 7B), just as in the case of FipA.

**Figure 7:** FtsZ is phosphorylated in a PknA-dependent manner. A. Purified FtsZ or its T343A mutant was phosphorylated by GST-PknA_13-273_ in the presence of [γ-^32^P] ATP followed by autoradiography. The lower blot is a Coomassie blue-stained gel showing the levels of FtsZ. B. Conditional knockdown of *pknA* was induced by growing *M. smegmatis* expressing an antisense construct of *pknA* (under the control of an acetamide-inducible promoter) in the absence (-) or in the presence (+) of acetamide for 12 h. Cells were lysed and lysates were immunoprecipitated with preimmune sera (first lane) or anti-FtsZ antibody, followed by immunoblotting with anti-phosphothreonine and reprobing with anti-FtsZ antibody. Blots shown are representative of three separate experiments.

### Formation of a Complex between FtsZ, FipA and FtsQ and the Role of PknA

Considering that FipA appeared likely to play a role in cell division, we tested whether FipA influences interaction of FtsZ with any divisomal protein which follows it to the site of division. Among the proteins which have been recognized as following FtsZ and preceding FtsW to the site of division is FtsQ of *E. coli* (or DivIB of *B. subtilis*). The ORFs Rv2151c and MSMEG_4229 (Figure S5) encode *M. tuberculosis* and *M. smegmatis* FtsQ respectively [30]. Like FtsZ, both FipA and FtsQ localize to mid-cell in dividing *M. smegmatis* (Figure S6) as observed by immunofluorescence microscopy. Numerical data show that FipA localizes to the septum to a similar extent in untreated and H_2_O_2_-treated cells (Table 2).

**Table 2:** Localization of FipA in *M. smegmatis*.

Growth condition	Septum	Poles	ND*
Untreated	52	9	39
Subjected to H_2_O_2_ stress	48	10	42

In each set, FipA localization was counted among 100 cells.

*Not determined.

We tested the possibility that FipA is part of a larger divisomal complex including FtsQ and FtsZ. FtsQ could be pulled down in a complex with FtsZ in wild type *M. smegmatis* as well as in FipA-KO (Fig. 8A) in the absence of stress. However, under H_2_O_2_ stress, FtsQ immunoprecipitated with FtsZ only in the wild type, but not in FipA-KO (Fig. 8A), suggesting that FipA is required for FtsZ to interact with FtsQ in oxidatively stressed cells, whereas FipA likely plays a redundant role in the absence of oxidative stress. In support of this contention, FipA-KO complemented with *fipA*_MTB_ rescued the ability of FtsZ to interact with FtsQ under oxidative stress (Fig. 8A). FtsZ-FtsQ interaction was compromised in oxidatively stressed cells of FipA-KO complemented with *fipA*_MTB(T77A)_ (i.e. phosphorylation-defective FipA) (Fig. 8B). Under oxidative stress, 67% of the FipA-KO cells showed punctate distribution of FtsQ in membranes with no visible localization at mid-cell, as opposed to 52% of the wild type cells showing septal localization of FtsQ (Table 3). Taken together, these results suggest that (a) FipA supports septal localization of FtsQ even under oxidative stress and (b) phosphorylation of FipA is required for FipA to fulfill this function.

**Figure 8:** Interactions between FtsZ, FtsQ and FipA *in vivo*. A. *M. smegmatis* wild type (WT) or FipA -KO (KO) or FipA -KO complemented with *fipA*_MTB_ (complemented) was left untreated (−) or treated (+) with H_2_O_2_, as described under “Materials and Methods”, lysed and immunoprecipitated with preimmune sera (first lane) or with anti-FtsZ antibody followed by immunoblotting with anti-FtsQ antibody. B. FipA-KO or FipA-KO complemented with *fipA*_MTB_(WT) or the T77A mutant, was grown, subjected to oxidative stress, lysed and immunoprecipitated with anti-FtsZ antibody followed by immunblotting with anti-FtsQ antibody. C. *M. smegmatis* strains mc^2^155, F1 or F2, were grown and subjected to the same treatment as in panel B, followed by immunoprecipitation with anti-His antibody (for pull down of FtsZ) and immunoblotting with anti-FtsQ antibody. D. *M. smegmatis* before or after conditional knockdown of *pknA* (performed as described under Fig. 7), was subjected to oxidative stress, lysed and immunoprecipitated with preimmune sera (first lane) or anti-FtsZ antibody, followed by immunblotting with anti-FtsQ antibody. E. *M. smegmati*s-F1 or -F2 cells subjected to oxidative stress, were lysed and immunoprecipitated with anti-His antibody followed by immunoblotting with anti-FipA antibody. Blots (A–E) were reprobed with anti-FtsZ antibody. Blots shown are representative of three separate experiments.

**Table 3:** Localization of FtsQ in FipA-KO and complemented strains.

Cell type and treatment	punctate *	septum	poles	ND**
WT (−) stress	13	64	21	2
WT (+)stress	30	52	13	5
KO (−)stress	19	58	19	4
KO (+)stress	67	0	3	30
KO with *fipA*_MTB_ (−) stress	15	61	15	9
KO with *fipA*_MTB_ (+) stress	35	45	12	8

*Cells showing punctate distribution of FtsQ in the membrane.

**Not determined.

In each set, FtsQ localization was scored in 100 cells.

In order to understand the role of phosphorylation of FtsZ on its interaction with FtsQ, merodiploid strains lacking the chromosomal copy of *ftsZ* and carrying an integrated copy of the wild type His-*ftsZ*_MTB_ (*M. smegmatis*-F1) or its T343A mutant (*M. smegmatis*-F2), were generated. FtsZ-FtsQ interactions were supported under oxidative stress by *M. smegmatis* strain F1 but not strain F2 (Fig. 8C). In *M. smegmatis*-F1, FtsQ showed septal localization in 67 and 55% cells in the absence of stress or under oxidative stress, respectively (Table 4). On the other hand, in *M. smegmatis*-F2, septal localization of FtsQ was visible in the absence of stress, but not in oxidatively stressed cells (Table 4). These observations suggest that phosphorylation of FtsZ is required for the interaction between FtsZ and FtsQ as well as for the septal localization of FtsQ. A role of PknA-mediated phosphorylation of FipA and FtsZ in sustaining FtsZ-FtsQ interactions under oxidative stress was also suggested by the observation that immunoprecipitation of FtsZ failed to pull down FtsQ in *pknA*-depleted cells (Fig. 8D) under oxidative stress. Further, immunoprecipitation of FtsZ from lysates of *M. smegmatis-*F1 or *M. smegmatis*-F2 strains showed that, like FtsQ, FipA could also be pulled down with wild type FtsZ_MTB_ but not with FtsZ_MTB(T343A)_ (Fig. 8E) under oxidative stress, suggesting that FtsZ phosphorylation is required for the FtsZ-FipA interaction.

**Table 4:** Localization of FtsQ in *M. smegmatis*-F1 and *M. smegmatis*-F2.

Cell type and treatment	punctate *	septum	poles	ND**
*M. smegmatis*-F1 (−) stress	19	67	7	7
*M. smegmatis*-F1 (+)stress	29	55	10	6
*M. smegmatis*-F2 (−)stress	26	53	13	8
*M. smegmatis*-F2 (+) stress	64	0	8	28

*Cells showing punctate distribution of FtsQ in the membrane.

**Not determined.

In each set, FtsQ localization was scored in 100 cells.

Immunoprecipitation of cell lysates with anti-FipA antibody, followed by immunoblotting with either anti-FtsQ or anti-FtsZ antibody showed that FipA could pull down FtsQ (Fig. 9A) or FtsZ (Fig. 9B) under oxidative stress However, FipA-FtsQ or FipA-FtsZ interaction was abrogated when *pknA* had been knocked down (Fig. 9A,B) supporting the contention that formation of the FtsZ-FtsQ-FipA complex under oxidative stress requires PknA. Taken together, our results suggest a role of PknA-mediated phosphorylation of FipA on T77 and FtsZ on T343 in mediating formation of a complex between FtsZ, FtsQ and FipA as well as their localization at mid-cell, under oxidative stress.

**Figure 9:** FipA is a bridging partner for interactions between FtsZ and FtsQ. A, B. *M. smegmatis* before or after conditional knockdown of *pknA*, was subjected to oxidative stress, lysed and immunoprecipitated with preimmune sera (lane 1) or anti-FipA antibody (lanes 2 and 3), followed by immunblotting with anti-FtsQ (A) or –FtsZ (B) antibody and reprobing with anti-FipA antibody. C. Recombinant S-tagged FtsQ_MTB_ immobilized on S-agarose was incubated with buffer only (lane 1) or with recombinant FipA_MTB_ followed by washing and further incubation with FtsZ_MTB_ (lane 2); or incubated with FipA_MTB_ and FtsZ_MTB_ simultaneously (lane 3). Resin-bound proteins were separated by SDS-PAGE and immunblotted with different antibodies as indicated. For lanes 4 and 5, Ni^2+^ -NTA bound His-tagged FtsZ_MTB_ was incubated with (lane 4) or without (lane 5) FipA_MTB_ followed by washing and further incubation with FtsQ_MTB_. Bound proteins were identified by immunoblotting with the indicated antibodies. The blot was reprobed with anti-FtsZ antibody. Blots shown are representative of three separate experiments.

Given the above findings, we tested the hypothesis that FtsZ, FtsQ and FipA are capable of forming a ternary complex *in vitro*. S-tagged FtsQ_MTB_ was immobilized on S-agarose, followed by simultaneous incubation with phosphorylated His-FtsZ_MTB_ and phosphorylated His-FipA_MTB_. The pulled down proteins were separated by SDS-PAGE and probed by Western blotting with anti -FtsZ and -FipA. Both FtsZ_MTB_ and FipA_MTB_ were pulled down from lysates (Fig. 9C, lane 3). When FipA_MTB_ was incubated with immobilized FtsQ_MTB_, beads were washed, and FtsZ_MTB_ was subsequently added, neither FipA_MTB_ nor FtsZ_MTB_ could be pulled down with FtsQ_MTB_ (Fig. 9C, lane 2). These observations suggest that prior interaction between FtsZ and FipA is necessary for formation of the FtsZ-FipA-FtsQ ternary complex. In support of this, FtsZ immunoprecipitates which contained FipA were able to pull down FtsQ (Fig. 9C, lane 4), whereas FtsZ immunoprecipitates alone could not pull down FtsQ (Fig. 9C, lane 5). These results suggest that FipA influences the ability of FtsZ to interact with partner divisomal proteins, and that initial interaction between FtsZ and FipA is necessary for ternary FtsZ-FipA-FtsQ complex formation.

## Discussion

The gene cluster encompassing the products of the ORFs *Rv0014c-Rv0019c* is conserved throughout the genus *Mycobacterium*. It encompasses two transmembrane sensor kinases PknA and PknB, a phosphatase PstP, a transpeptidase PBPA and the FHA domain protein encoded by *Rv0019c* (FipA). There has been speculation that this gene cluster plays a role in cell division [31]. However, knowledge of the roles of the individual gene products of this cluster in the genus *Mycobacterium*, is scanty. The *dcw* cluster is conserved across the genus mycobacterium and includes genes such as *ftsZ*, *ftsQ* and *ftsW* whose products are central to the process of cell division. Here we establish two important findings. In the first instance we demonstrate a synergy of action between two products of the first gene cluster, (PknA and the FHA domain protein FipA), and two products of the *dcw* cluster (FtsZ and FtsQ) in maintaining cells in a division-competent state under oxidative stress. We uncover a novel role of phosphorylated FipA in assembly of the divisome under oxidative stress. In the second instance, we demonstrate that the network of interactions between FtsZ, FipA and FtsQ, is critically dependent on the serine/threonine kinase PknA. These findings are discussed below.

*M. tuberculosis* resides within host macrophages following inhalation into the alveolar spaces of the lung. The bacterium is exposed to adverse environmental conditions and toxic agents such as reactive oxygen intermediates (ROI). It is logical that the bacterium must be endowed with mechanisms of withstanding the stressful conditions of its intracellular niche to an extent that allows multiplication and survival within macrophages. Control of cell division as well as maintenance of cell shape are critical factors for the survival of mycobacteria within the host. After replication, the multiprotein complex that comprises the divisome, assembles at mid-cell in order to facilitate cell division [32]. In mycobacteria, the repertoire of proteins required for cell division of mycobacteria within macrophages, remains incompletely understood. In order to test whether the FHA domain protein FipA plays a role in supporting intramacrophage growth of *M. tuberculosis*, *fipA* was knocked down. Knockdown of *fipA* was associated with a cell division defect of *M. tuberculosis* in macrophages after 5 days of infection, providing evidence that FipA is required to sustain growth of *M. tuberculosis* within macrophages. The role of FipA was investigated using *M. smegmatis* as the model. Knockout of *fipA* resulted in a cell division defect in *M. smegmatis* exposed to H_2_O_2_. In *E. coli*, cell division block is frequently associated with induction of *recA*-dependent SOS response [33]. In *M. tuberculosis*, ROI produced by macrophages can damage DNA and induce the SOS response. In the classical pathway, DNA damage induces *recA* and *lexA*-dependent SOS response [34]. However, in this instance we could rule out the possibility of induction of a classical SOS response at the concentrations and times of H_2_O_2_ exposure used. Consequently, we investigated other causes of FipA-linked cell division block under oxidative stress, focusing on the interaction of FipA with well-characterized proteins of the divisome.

Our results indicate that FipA interacts with FtsZ in a phosphorylation-dependent manner. Earlier studies have focused on biochemical characterization of PknA [35], and identified substrates such as MurD [36]. Kang *et al*. [20] reported that in mycobacteria, partial knock down of *pknA* or *pknB* leads to the formation of narrow and elongated cells, suggesting a role of these protein kinases in cell division. However, the significance of PknA-dependent phosphorylation of divisomal proteins is still not clear. Unlike Thakur and Chakraborti [35] we did not observe phosphorylation-dependent inhibition of the GTPase activity of FtsZ. It is pertinent to point out that Thakur and Chakraborti [35] used GST-FtsZ, whereas we have worked with His-FtsZ. It may be mentioned that Schulz *et al*. [37] failed to observe PknA-dependent inhibition of polymerization of *Corynebacterium glutamicum* FtsZ. During infection, membrane-bound kinases are thought to transmit environmental signals inside bacteria. In fact, *pknA* and *pknB* are upregulated by more than 10-fold when THP-1 cells are infected with *M. tuberculosis* [38]. It therefore appears likely that the serine/threonine kinases of mycobacteria play important roles during infection. Understanding their function could in the long run provide newer directions for development of antituberculosis drugs. With this in view, we pursued investigation on the possible role of PknA in cell division. We now establish that FipA is phosphorylated on T77 in a PknA-dependent manner, and elucidate a functional role for such a phosphorylation event. Coimmunoprecipitation assays confirm that the FHA domain of FipA is necessary for its interaction with PknA. FipA_MTB_ could complement FipA-KO with restoration of growth and survival under oxidative stress. The phosphorylation-defective T77A mutant failed to support cell division in FipA-KO under oxidative stress, underscoring the importance of PknA-dependent phosphorylation of FipA in sustaining cell division under oxidative stress.

In *E. coli*, FtsQ interacts with a large number of divisomal proteins [39] and is required for divisome assembly [40]. Recruitment of FtsZ, FtsQ and FtsA to mid-cell is required for the septal localization of FtsW [41]. In mycobacteria, FtsQ is required for localization of FtsW to the septum in dividing cells (unpublished observations) suggesting that it plays an important role in mycobacterial cell division. We provide evidence that FipA interacts with FtsZ and FtsQ in a PknA-dependent manner. We hypothesize that FipA is required for divisomal protein assembly under oxidative stress, in a manner that is dependent on phosphorylation of FipA mediated by PknA. We show that in the absence of oxidative stress, FtsQ interacts with FtsZ *in vivo* both in the wild type as well as in FipA-KO, although the two proteins do not interact directly with each other (Fig. 9C). This suggests that FipA, as a member of the divisomal complex, plays a redundant role in the absence of stress. Additional, unidentified accessory protein(s) probably fulfill a bridging function (between FtsZ and FtsQ) under normal conditions. This probably suffices to sustain septation of growing cells even in the absence of FipA. However, the accessory protein(s) are probably incapable of functioning under oxidative stress. FipA assumes a critical role in these conditions. In vitro grown *M. smegmatis* exposed to H_2_O_2_ or *M. tuberculosis* growing in macrophages, are longer than cells cultured *in vitro* in the absence of exogenous oxidative stress. These cells nevertheless survive in the presence of functional FipA. On the other hand, there is a much more severe division block under these conditions in the absence of FipA. It therefore seems reasonable to contend that FipA supports cell division in *M. tuberculosis* growing in macrophages to an extent that is optimal for its survival in the stressful environment of the phagosome. The FipA proteins are unique to mycobacteria, even though FtsZ and FtsQ are present across numerous genera. It is likely that FipA fulfils a function in the process of cell division and multiplication, specifically required for survival of mycobacteria in the intracellular mileu of the host. Our observations provide knowledge for the first time that in mycobacteria (i) there is synergy between the gene cluster Rv0014c-Rv0019c and the *dcw* cluster; (ii) PknA-dependent phosphorylation events fine tune cell division and play a critical role under oxidative stress and (iii) the product of the ORF *Rv0019c*, FipA, plays an important role in supporting cell division under oxidative stress. While our work was in progress, Gupta *et al*. [42] reported that FipA (Rv0019c) interacts with polyketide-associated protein, PapA5 of *M. tuberculosis in vitro* and that it is phosphorylated by PknB on T36. However, the physiological importance of these findings is unclear in the absence of any in vivo experiments. It remains to be investigated whether PknA-mediated phosphorylation of FipA on T77 and PknB-mediated phosphorylation on T36 are interdependent, whether PknB-dependent phosphorylation is constitutive or inducible, and whether it too plays a role in cell division. It is possible that site-specific phosphorylations of FipA by two different kinases regulate interaction with different substrates. Another FHA domain containing protein, GarA [43] has been found to be phosphorylated by two kinases, PknG and PknB which differentially regulate its interaction with other proteins. Detailed investigations to resolve these unanswered question are in progress. In summary, our observations offer new insight into how targeting FtsZ-FipA interaction could block cell division to an extent that would compromise mycobacterial multiplication in macrophages.

## Materials and Methods

### Molecular Biological Procedures

Standard procedures for cloning and analysis of DNA, PCR, electroporation and transformation were used. Enzymes used to manipulate DNA were from Roche Applied Science, Mannheim, Germany. All constructs made by PCR were sequenced to verify their integrity. *E. coli* strains were routinely grown in Luria broth (LB). Details of strains and plasmids are provided in Table S1.

### Construction of Suicidal Delivery Vector for Inactivation of fipA in *M. smegmatis*

The two step homologous recombination strategy described by Parish and Stoker [44] was used to disrupt *MSMEG_*0034, the counterpart of *Rv0019c* at its native locus in *M. smegmatis*. Briefly, a suicide plasmid was constructed in three steps. First, an 860 bp DNA fragment containing the 5′ end of *MSMEG_0034* alongwith upstream sequence was PCR amplified using the genomic DNA of wild type *M. smegmatis* mc^2^155 as template and the primer pair FipA 1F sense and FipA 1F antisense (Table S2). The amplicon was cloned between the asymmetric *Hind*III and *Bam*HI sites of p2NIL to give pJB110. In the next step, a 900 bp fragment bearing the 3′ end of *MSMEG_0034* and its downstream region was amplified using the primer pair FipA 2F sense and FipA 2F antisense (Table S2) and cloned between the *Bam*HI and *Pac*I sites of pJB110 to give pJB111 carrying a truncated *fipA* gene. The hygromycin cassette was excised from pUC-HY–INT (Mahenthiralingam *et al.*, 1998) and introduced into pJB111 to give pJB112. Finally, a 6.1 kb *Pac*I cassette carrying the *lacZ*, *aph* and *sacB* genes, was isolated from pGOAL17 and inserted into pJB112 to generate the suicide plasmid pJB113.

### Isolation of the FipA –Knockout Mutant

Denatured pJB113 was electroporated into electrocompetent cells of *M. smegmatis* mc^2^155. Cells were plated on Lemco agar supplemented with hygromycin B, kanamycin and 50 µg/ml x-gal. Blue colonies were streaked onto Lemco agar without any selection to enhance the recombination process. Cells were then plated onto Lemco agar supplemented with 2% sucrose and 50 µg/ml x-gal. The white colonies were restreaked onto replica plates containing hygromycin, x-gal and sucrose, either without or with kanamycin. White, kan^S^, hyg^R^, suc^R^ colonies generated by double crossover represented the *fipA* –inactivated strain (FipA–KO). Expression of FipA was checked using antibody raised against FipA.

### Complementation of FipA_MTB_ in FipA-KO Using an Integrating Vector

An integrating vector carrying *His-FipA*(or its mutants) of *M. tuberculosis* under the control of the *hsp60* promoter was constructed as described earlier [19]. Complementation with *fipA*_MTB_ was achieved by electroporation of the integrating vector into FipA–KO. The presence of His-FipA was confirmed by Western blotting using anti-His antibodies.

### Cloning and Expression of *M. tuberculosis* H37Rv Genes

*FipA* was amplified from genomic DNA of *M. tuberculosis* H37Rv using the sense primer “a” and antisense primers “d” (for pET28a+) and “e” (for pET29a+) depicted in Table S2. The amplicons were cloned between asymmetric *Bam*HI and *Hind*III sites in pET28a or the *Bam*HI and *Eco*RI sites in pET29a+ to generate pJB120 and pJB121 respectively. *E. coli* C41 (DE3) harbouring the respective constructs was grown to an Abs_600_ of 0.6 at 37^o^C, IPTG was added at a concentration of 0.25 mM, and growth was continued for 2–3 h. His- or S-tagged proteins were purified from cell lysates by chromatography on Ni^2+^-NTA- or S-agarose respectively. Mutants of FipA_MTB_ were generated by overlap extension PCR. Initial rounds of PCR were performed using primers “a”and “b”; or primers “c” and “d” (or “e”) (Table S2). Using the products of the initial round as template, the second round of PCR was performed using primers “a” and “d” (or “e”). Products were cloned in pET28a+ or pET29a+. The T343A mutant of FtsZ was generated using pJB101 (Datta *et al*., 2002) as template and primers “a” and “d” (Table S2).

*ftsQ* was amplified using the sense and antisense primers shown in Table S2, and cloned either in pET28a+ or in pET29a+ between the *Bam*HI and *Hind*III sites. Expression was carried out in *E. coli* C41(DE3) using 0.1 mM IPTG for 4 h at 37°C.

The kinase domain of *pknA* (*pknA*_13-273_) was amplified using the sense and antisense primers shown in Table S2, and cloned between the *Bam*HI and *Eco*RI sites of pGEX-2T to generate the plasmid pJB122. Expression was carried out in *E. coli* BL21 by induction with 0.1 mM IPTG at 37°C for 4 h, and the expressed protein was purified by chromatography on glutathione Sepharose. The K42A mutant was generated by overlap extension PCR using primers “b” and “c” depicted in Table S2. His-PknB_1–276_ was purified as described earlier [19]. The *pstP* (Rv0018c) gene was amplified using the sense and antisense primer pair shown in Table S2, and cloned between the *Bam*HI and *Hind*III sites of pET29a^+^. N-terminal S-tagged PstP was obtained by induction for 3 h at 37°C with 50 µM IPTG and purified by chromatography on S-agarose

### Construction of ftsZ Replacement Vectors in *M. smegmatis*

A construct for replacement of the chromosomal *ftsZ* of *M. smegmatis* was generated using the method of described above [44]. A suicide plasmid with a 488 bp internal deletion in the *ftsZ* gene was constructed in two steps. In the first step, a 1244 bp DNA fragment encompassing the 5′ end of *ftsZ* and its upstream region was PCR amplified using the primer pair FtsZ 1F sense and FtsZ 1F antisense (Table S2) and cloned in pBluescript SK between the asymmetric *Bam*HI and *Eco*RI sites to give rise to pJB114. In the next step 1153 bp of DNA bearing the 3′ end of *ftsZ* and its downstream flanking region was amplified using the primer pair FtsZ 2F sense and FtsZ 2F antisense (Table S2) and cloned between the *Eco*RI and *Hind* III sites of pJB114 to generate pJB115. The truncated *ftsZ* gene was excised from pJB115 by digesting with *Bam*HI and *Hind*III and cloned into p2NIL between the same sites to generate pJB116. Finally, the 6.1 kb PacI fragment was isolated from pGOAL19 and inserted into pJB116 to generate the suicide plasmid pJB117.

### Isolation of *M. smegmatis* Strains Carrying Wild Type or Mutated ftsZ_MTB_

*M. smegmatis* was electroporated with denatured pJB117. Single cross over (SCO)s were selected on agar plates containing kanamycin and x-gal. Kanamycin-resistant blue SCOs were isolated. In the next step, His-tagged *ftsZ*_MTB_ (or its mutant) was cloned under the control of the *hsp60* promoter in pUC19 using *Kpn*I and *Hind*III sites as described above. The 3.757kb Hyg-integrase cassette was excised from pUC-HY-INT [45] and inserted into the above construct to generate an integrating vector. Before inactivation of *ftsZ* at its native location, *ftsZ*_MTB_ in the integrating vector was electroporated into the SCOs. The resultant merodiploid strains carrying His-tagged *ftsZ*_MTB_ (*M. smegmatis*-F1) or *ftsZ*_MTB(T343A)_ (*M. smegmatis*-F2) were then screened for double cross over (DCO) as described earlier [46]. White kan^S^ Hyg^S^ and sucrose-resistant DCOs were analyzed by PCR.

### *In Vitro* Kinase Assay

In vitro kinase assays were performed with the purified kinase domain of PknA_13–273_ (1 µg) in 25 mM Tris/HCl, pH 7.5, 5 mM β-glycerophosphate, 2 mM DTT, 2 mM MnCl_2_, 0.1 mM sodium orthovanadate as described by Dasgupta *et al*. (2006). Dephosphorylation assays were carried out in 50 mM HEPES buffer pH 7.5 containing 0.1 mM EDTA, 1 mM DTT and 5 mM MnCl_2_ as described earlier [19]. In some experiments, proteins separated by SDS-PAGE were electrotransferred and Western blotting was performed using monoclonal anti-phospho-threonine or anti-phosphoserine (Sigma Chemical Co.) or anti-phospho-tyrosine (Cell Signaling Technology) antibody.

### Conditional Inactivation of pknA in Mycobacteria

The *pknA* gene was amplified using the primer pair pknA sense and pknA antisense (Table S1) followed by cloning of the PCR product in reverse orientation in the vector pSD29 [47] between the *Bam*HI and *Eco*RV sites to generate pJB118. In order to conditionally inactivate *pknA*, *M. smegmatis* was electroporated with pJB118. Transformants were grown up to mid log phase and induced with 0.2% acetamide for different periods of time. Western blotting was performed to confirm the antisensing of PknA.

### Knock Down of FipA in *M. tuberculosis*

For knock down of *fipA*_MTB_, an antisense construct (pJB119) of *fipA* was generated by PCR amplification of the *fipA* gene using the primer pair FipA_MTB_ sense and FipA_MTB_ antisense (Table S2) followed by cloning of the PCR product in reverse orientation under the control of the *hsp60* promoter using the strategy described by Sureka *et al.* [48]. Western blotting using anti-FipA antibody was performed to confirm the antisensing of *fipA*.

### Induction of Oxidative Stress and Treatment with Mitomycin C

Cells were subjected to H_2_O_2_-mediated oxidative stress as described earlier [48]. Briefly, cells were grown to an OD_600_ of 0.3 to 0.4, diluted into fresh medium to an OD_600_ of 0.2 and treated with 50 µM hydrogen peroxide for 1 h, followed by addition of hydrogen peroxide to 5 mM and incubation for the desired period of time. Mitomycin C treatment was carried out similarly by exposing cells (suspended at an OD_600_ of 0.2) to mitomycin C (0.2 µg/ml) for 4 h.

### Preparation of Cell Lysate, Antibodies and Immunoprecipitations

Cell lysates were prepared by disrupting cells in a Mini Bead Beater (Biospec Products) as described earlier [48]. Immunoprecipitations were carried out by overnight incubation of lysates with antibodies at a dilution of 1∶1,000 at 4°C, followed by precipitation with Protein A/G agarose for 3 h. Antibodies against the kinase domain of PknA, PknB, PBPA, PstP, FtsQ, FipA and FtsZ were raised by Imgenex, Bhubaneswar.

### Fluorescence Microscopy

Immunostaining was performed as described earlier [14]. Briefly, cells were fixed by incubation for 15 minutes at room temperature followed by 45 minutes on ice in 2.5% (v/v) paraformaldehyde, 0.04% (v/v) glutaraldehyde, 30 mM sodium phosphate (pH 7.5). After washing in PBS, the cells were permeabilized by exposing to 2% toluene for 2 min, and immediately transferred to slides. The slides were washed with PBS, air-dried, dipped in methanol (−20°C) for 5 min and then in acetone (−20°C) for 30 s and allowed to dry. After rehydration with PBS, the slides were blocked for 2 h at room temperature with 2% (w/v) BSA-PBS and incubated for 1 h with appropriate dilutions of primary antibody in BSA-PBS. The slides were washed extensively with PBS and then incubated with a 1∶1,000 dilution of Alexa 488-conjugated anti-rabbit IgG (Molecular Probes, Eugene, OR, USA) in BSA-PBS. After extensive washing with PBS, the slides were mounted using 50% glycerol. In controls for assessing specificity of the primary antibodies, the incubation with the preimmune sera was included. Images were viewed in a Zeiss Axioimager A1 microscope.

## Supporting Information

Figure S1 A. Schematic representation of the genomic region of *M. tuberculosis* encompassing Rv0014c-Rv0019c and the corresponding region in *M. smegmatis*. B. Alignment of the amino acid sequences of FipA of *M. tuberculosis* (encoded by Rv0019c) and *M. smegmatis* (encoded by MSMEG_0034). The FHA domain is over-scored.
(0.21 MB JPG)

Figure S2 A. Expression of PknB, PknA, PBPA, PstP, FipA and FtsZ in wild type (WT) or FipA-KO (KO) or FipA-KO complemented with fipA of *M. tuberculosis* (com.). B,C. Transcriptional analysis of lexA and recA in *M. smegmatis*. Cells were treated with hydrogen peroxide or mitomycin C. RNA was isolated and subjected to q-RT-PCR for the lexA (B) and recA (C) genes. Fold increase represents the change with respect to untreated cells. Values shown are means with S.D. of three separate determinations.
(0.11 MB JPG)

Figure S3 Mass analysis of FipA or FipA phosphorylated by PknA.
(1.82 MB TIF)

Figure S4 Mass analysis of FtsZ (unphosphorylated), or phosphorylated by PknA or FtsZ(T343A).
(0.47 MB TIF)

Figure S5 Schematic representation of the genomic region encompassing the dcw cluster of *M. tuberculosis* (Mtb) and *M. smegmatis* (Msmeg).
(1.27 MB TIF)

Figure S6 Immunolocalization of FipA (A) and FtsQ (B) in *M. smegmatis*. Immunolocalization of was carried out by incubation with anti-FipA or anti-FtsQ antibody followed by staining with Alexa 488-conjugated rabbit IgG and visualization by fluorescence microscopy.
(0.03 MB JPG)

Table S1 List of strains and plasmids used in this study.
(0.04 MB DOC)

Table S2 Primers used in this study.
(0.06 MB DOC)
